# Identification of Significant Genes and Pathways for the Chronic and Subacute Cutaneous Lupus Erythematosus via Bioinformatics Analysis

**DOI:** 10.1155/2022/9891299

**Published:** 2022-09-29

**Authors:** Yan Teng, Sujing Li, Yang Ding, Yibin Fan, Miao He, Hengzhen Li, Xiaohua Tao, Youming Huang

**Affiliations:** ^1^Health Management Center, Department of Dermatology, Zhejiang Provincial People's Hospital, Affiliated People's Hospital of Hangzhou Medical College, Hangzhou 310014, China; ^2^Bengbu Medical College, Bengbu, China; ^3^Department of Orthopedics, Xiangya Hospital, Central South University, Changsha, 410008 Hunan, China

## Abstract

**Background:**

Chronic cutaneous lupus erythematosus (CCLE) and subacute cutaneous lupus erythematosus (SCLE) are both common variants of cutaneous lupus erythematosus (CLE) that mainly involve the skin and mucous membrane. Oral mucosal involvement is frequently observed in patients of CLE. Despite that they have different clinicopathological features, whether there is a significant difference in pathogenesis between them remains unclear. Herein, we investigated specific genes and pathways of SCLE and CCLE via bioinformatics analysis.

**Methods:**

Microarray expression datasets of GSE109248 and GSE112943 were both retrieved from the GEO database. Differentially expressed genes (DEGs) between CCLE or SCLE skin tissues and health controls were selected by GEO2R. Common DEGs were picked out via the Venn diagram software. Then, functional enrichment and PPI network analysis were conducted, and the top 10 key genes were identified via Cytohubba.

**Results:**

Totally, 176 DEGs of SCLE and 287 DEGs of CCLE were identified. The GO enrichment and KEGG analysis of DEGs of SCLE is significantly enriched in the response to virus, defense response to virus, response to IFN-gamma, cellular response to IFN-*γ*, type I IFN signaling pathway, chemokine activity, chemokine receptor binding, NOD-like receptor signaling pathway, etc. The GO enrichment and KEGG analysis of DEGs of CCLE is significantly enriched in the response to virus, regulation of multiorganism process, negative regulation of viral process, regulation of lymphocyte activation, chemokine receptor binding, CCR chemokine receptor binding, NOD-like receptor signaling pathway, etc. The top 10 hub genes of SCLE and CCLE, respectively, include STAT1, CXCL10, IRF7, ISG15, and RSAD2 and CXCL10, IRF7, IFIT3, CTLA4, and ISG15.

**Conclusion:**

Our finding suggests that SCLE and CCLE have the similar potential key genes and pathways and majority of them belong to IFN signatures and IFN signaling pathway. Besides, the NOD-like receptor signaling pathway might also have an essential role in the pathogenesis of SCLE and CCLE. Together, the identified genes and signaling pathways have enhanced our understanding of the mechanism underlying the occurrence and development of both SCLE and CCLE.

## 1. Introduction

Lupus erythematosus (LE), as a chronic autoimmune disorder, is induced by an interplay of genetic, hormonal, and environmental factors and characterized with a wide range of clinical forms from skin and mucosal lesions to life-threatening systemic manifestations. Oral involvement ranges from 9% to 45% in patients of SLE and 3% to 25% in patients of CLE [1, 2]. Among CLE patients, higher cutaneous disease activity might have a significant correlation with the following oral manifestations: discoid plaques, cobblestone, and red/brown-pigmented macules. Additionally, the presence of gingivitis was associated with systemic inflammation [3]. According to the clinical and histological features, CLE was generally categorized into acute CLE (ACLE), SCLE, and CCLE. The most common type of CCLE is discoid LE (DLE), which is characterized with erythema, telangiectasias, atrophy, and regression with scarring. Approximately 30% of DLE patients have the oral mucosal involvement. SCLE is characterized with annular and lesions in sun-exposed regions [4, 5]. Oral ulcers are the common clinical presentation. Above all, oral involvement acts as an indicative role to the diagnosis and evaluation of CLE disease course.

For the individuals with a genetic predisposition, multiple environmental factors can activate innate and adaptive immune responses that contribute to the formation of CLE skin lesions. There is strong evidence that clarifies the function of cytotoxic T cell-mediated immune response against the epidermis with the result of keratinocyte death and nuclear antigens release [6]. Thereby, B cells might act as antigen-presenting cells initiating the activation of autoreactive T cell [7]. Additionally, it has been suggested that keratinocytes themselves may be involved with the self-perpetuating cycle of lesions by producing type 1 and 2 IFN and IFN-regulated proinflammatory cytokines [8, 9].

SCLE and CCLE are the major two categories of CLE. Although they have different clinicopathological features, the specific pathogenesis of the two and whether there is a huge difference between them have not been completely clarified. Harrris et al. [10] have indicated that the gene expression of CLE subtypes differs from health control skin with the predominance of upregulated expression of type 1 IFN and T cell chemotactic genes. However, there is more similarity among the subtypes of CLE. In our study, we selected the gene microarray (GSE109248 and GSE112943) from the Gene Expression Omnibus databases (GEO) to screen and identify the DEGs of SCLE and CCLE compared with the healthy skin control. Then, enrichment analysis and protein-protein interaction (PPI) network analysis were performed to select possible pathways and key genes that participated into the pathogenesis of SCLE and CCLE. This study might provide a new understanding of pathogenesis of SCLE and CCLE.

## 2. Materials and Methods

### 2.1. Microarray Information

The microarray expression profiles of GSE109248 and GSE112943 were retrieved from NCBI-GEO (https://www.ncbi.nlm.nih.gov), a free public database of microarray profile. Titles related to SCLE and CCLE were screened, and the details were further evaluated. The datasets of GSE109248 and GSE112943 were both based on the GPL10558, Illumina HumanHT-12 V4.0 expression beadchip platform. GSE109248 collected 6 skin samples from the CCLE, 12 skin samples from the SCLE, and 14 control skin samples. GSE112943 collected 6 skin samples from the CCLE, 10 skin samples from the SCLE, and 10 control skin samples. The volcano plot analysis was performed by GraphPad Prism 9.0.

### 2.2. Data Processing of DEGs

The DEGs between CCLE and SCLE skin samples and skin control samples were identified via GEO2R online tool via the standard |LogFC| > 2 and adjusted *P* value < 0.05 [11]. Then, the raw data in TXT were processed in Venn software online to select the common DEGs of CCLE and SCLE among the two datasets.

### 2.3. GO Enrichment and KEGG Pathway Analysis

Gene ontology (GO) analysis is a commonly applied method to define genes and its RNA or protein product to identify unique biological properties of high-throughput transcriptome or genome data. The Kyoto Encyclopedia of Genes and Genomes (KEGG) analysis is a collection of datasets managing the genomes, diseases, biological pathways, drugs, and chemical materials. We utilize the Database for Annotation, Visualization, and Integrated Discovery (DAVID 6.8, https://david.ncifcrf.gov) to perform the GO analysis and KEGG analysis in helping classify the DEGs (*P* value < 0.05). The GO enrichment analysis comprises biological processes (BP), cellular components (CC), and molecular functions (MF).

### 2.4. PPI Network Formation and Identification of Key Genes

The PPI network of DEGs was created by Search Tool for the Retrieval of Interacting Genes (STRING; https://www.string-db.org). The top 10 hub genes were picked out via the Cytohubba, a plugin of Cytoscape software (Cytoscape, 3.9).

## 3. Results

### 3.1. Identification of DEGs in SCLE and CCLE

Through the GEO2R online tools, we picked out 288 DEGs of CCLE and 283 DEGs of SCLE from GSE109248 and 357 DEGs of SCLE from GSE112943 (Figure 1). Then, we utilized the Venn diagram software to select the common DEGs in the two categories of DEGs from GSE109248 and GSE112943. Results indicated that a summary of 176 commonly expressed DEGs of SCLE was identified (Figure 2). Then, we selected the 358 DEGs of SCLE from GSE112934 to perform the following analysis.

### 3.2. DEGs of GO and KEGG Pathway Analysis in SCLE and CCLE

288 DEGs of CCLE and 176 DEGs of SCLE were analyzed for GO and KEGG analysis by DAVID software. The BP, CC, and MF analysis indicated DEGs of defense response to virus, regulation of multiorganism process, negative regulation of viral process, regulation of lymphocyte activation, cornified envelope, secretory granule membrane, chemokine receptor binding, cytokine activity, CCR chemokine receptor binding, etc. The KEGG analysis indicated that DEGs of CCLE were significantly enriched in the viral protein interaction with cytokine and cytokine receptor, primary immunodeficiency, NOD-like receptor signaling pathway, etc. The BP and MF analysis demonstrated that DEGs of SCLE were significantly enriched in the response to virus, response to IFN-gamma, cellular response to interferon-gamma, type I interferon signaling pathway, MHC class I protein binding, chemokine activity, chemokine receptor binding, and MHC protein binding. The KEGG analysis showed that DEGs of SCLE were significantly enriched in the cytokine-cytokine receptor interaction, cytosolic DNA-sensing pathway, NOD-like receptor signaling pathway, etc. (Tables 1 and 2 and Figure 3).

### 3.3. PPI Network Analysis and Identification of Key Genes

The PPI network of DEGs was created by STRING to screen the most significant clusters of the DEGs. As revealed in Figures 4 and 5, a total of 171 nodes and 447 edges in the PPI network of DEGs of SCLE and 99 nodes and 629 edges in the PPI network of DEGs of CCLE were found. Cytohubba, a plugin Cytoscape, was performed to identify the hub genes in the DEGs. The top 10 hub genes were picked out. The top 10 hub genes of SCLE and CCLE, respectively, include STAT1, CXCL10, IRF7, ISG15, RSAD2, IFIT3, OASL, GBP1, OAS1, and OAS2 and CXCL10, IRF7, IFIT3, CTLA4, ISG15, OAS2, RASD2, CCL5, GBP1, and OAS1 (Tables 3 and 4).

## 4. Discussion

CCLE and SCLE are both common variants of CLE that may occur independently or as clinical manifestations of SLE [12, 13]. Concern about the appearance of cutaneous rashes leads majority of patients with DLE or SCLE to require effective treatment. Particularly, early treatment of DLE is essential to minimize the risk of skin scarring. A subset of patients fails to respond to classical therapies that include topical, intralesional, or systemic antimalarial therapy. Therefore, further understanding of the pathogenesis of the disease contributes to find a new breakthrough in the treatment. Additionally, even though CCLE and SCLE both belong to the CLE, they have different clinical manifestations and pathological changes. Whether there is a huge difference in pathogenesis between them remains to be further investigated.

The pathogenesis of SLE is multifactorial always with the abnormal expression of molecules that are associated with the type I IFN signaling pathway [14]. In our study, the results of GO analysis revealed that the DEGs of SCLE were primarily enriched in the response to IFN-gamma, cellular response to IFN-gamma, and type I IFN signaling pathway. Inappropriate activation of IFN family IFN and its immune regulatory pathway might act a significant role in the formation of LE as well as CLE. In skin disease of LE, the type I IFNs are believed to participate in amplifying the lesional inflammation by eliciting the IFN-inducible chemokines and recruiting potentially autoreactive T cells into skin lesions. Additionally, interplays between the chemokine receptor CXCR3 and its IFN-inducible ligands CXCL9 and CXCL10 induce lesional inflammation in this condition. This is consistent with our results that the top 10 hub genes of SCLE and CCLE both include CXCL10 [15, 16]. Increasing evidence has recognized the anti-type I IFN receptor antibodies as a therapeutic strategy for the clinical treatment of SLE. Nico et al. once clarified the identity and similarities between skin and oral lesions and also demonstrated that oral LE was characterized with stronger expression of IFN-gamma [17, 18]. Above all, they might become a promising therapy to manage CLE, oral LE, and skin and/or oral involvement of SLE.

Additionally, the result of our study demonstrated that the top 10 genes of CCLE and SCLE mostly overlap that include CXCL10, IRF7, ISG15, OAS1, OAS2, RASD2, GBP, and IFIT3. 2′-5′-Oligoadenylate synthetase (OAS), a type of important antiviral proteins, is induced by IFN. The OAS gene family includes OAS1, OAS2, OAS3, and OASL genes, which have similar structure and function. OAS1, OAS2, and OASL were all found to be significantly overexpressed in PBMC of SLE using gene microarray. Moreover, their expression was supposed to become the indicators of disease activity of SLE [19]. Interferon-stimulated gene 15 (ISG15), an ubiquitin-like protein, is one of the IFN-inducible gene signatures. ISG15 also participated in the pathogenesis of SLE and is correlated with the disease activity at baseline [20]. Braunstein et al. [21] reported that OAS1, OASL, and ISG15 were found to have an increase in SCLE and DLE regardless of concomitant SLE.

Interferon regulatory factor 7 (IRF7) is a type I IFN-dependent key transcriptional regulator of immune responses and is present in an inactive form in the cytoplasm of normal cells when viruses infect cells. Although increasing studies have confirmed the function and role of genetic polymorphism of IRF7 gene in the formation of SLE, more researches are acquired in the human body to further clarify the precise relationship between IRF7 and SLE [22, 23]. Radical S-adenosyl methionine domain-containing 2 (RSAD2) is a host protein with extensive antiviral activity. Previous studies have shown that RSAD2 is closely correlated with the immune response. Further qRT-PCR verification in mouse B lymphocytes showed that RSAD2 was still significantly upregulated in SLE B lymphocytes compared with normal mouse B lymphocytes [24, 25]. The large GTPase human guanylate-binding protein 1 (GBP1) is a pivotal mediator of angiostatin effects of inflammation and is elicited by IFN-*α* and IFN-*γ* in endothelial cells (ECs). The relationship between GBP1 and LE is rarely reported. Similar to our study, a bioinformatics analysis conducted by Liu et al. [26] also found that GBP1 is one of the top 10 hub genes of SLE. Interferon (IFN) inducible gene 3 (IFIT3) is also elevated in SLE. Wang et al. [27] proposed that IFIT3 is one of the genes that elicits the cGAS-STING signaling pathway in SLE monocytes to be overactive. It may be acted as a treatment target to stop the type I IFN and other proinflammatory cytokine production via the cGAS-STING signaling pathway. However, the genes mentioned above have not been reported to have relationship with CLE that needs more studies.

The GO analysis of DEGs with SCLE and CCLE both indicated that the DEGs were mostly enriched into the chemokine receptor binding and NOD-like receptor signaling pathway. Chemokines are a category of chemotactic cytokines that participate in immune and inflammatory responses through the chemoattraction and leukocyte activation. Except CXCL9 and CXCL10 mentioned above, other members of the chemokine family include CXCR2, CXCR3, CXCR5, CCR2, CCR6, CCL2, and CCL17 that were also reported to have abnormal expression in CLE [28]. NOD-like receptors (NLRs) are an evolutionarily conserved family of innate immune receptors that were initially supposed to be responsive to intracellular pathogens (bacterial wall components, damaged membrane, toxins, uric acids, etc.) and endogenous byproducts of tissue damage. Recently, some studies have revealed that NLRs also act crucial roles in various biological processes like the antigen presentation regulation, inflammatory responses, embryonic development, and cell death. Various types of immune cells like dendritic cells, macrophages, B lymphocytes, and T lymphocytes all have expressed NOD2. Researches investigating the expression and function of NOD2 in SLE are relatively rare [29]. Yu et al. [30] indicated that compared with healthy controls the expression of NOD2 in plasmacytoid dendritic cells and monocytes of SLE patients was greatly increased. Bacterial exposure increased the expression of NOD2 in monocytes contributing to proinflammatory cytokine production by PBMCs that aggravated the condition of SLE. However, the limitations of our study could not be ignored. Firstly, some other important factors including age, race, and regions should be considered as well. Additionally, the potential key genes need further experimental verification by RT-qPCR in clinical samples, contributing to the final conclusions just speculative. Finally, the specific mechanisms in which these crucial genes play are not completely clarified that need more evidence.

## 5. Conclusions

The top hub genes of both CCLE and SCLE are almost induced by IFN, which support the significant role of IFN gene signatures and IFN signaling pathway in CLE. However, the hub genes like IRF7, IFIT3, and GBP1 are only reported to be related to SLE but not CLE. Although the hub genes like OAS1, OASL, and ISG15 and chemokine like CXCL10 are reported to have an abnormal expression in CLE, the specific roles of them in the pathogenesis of CLE are still not clarified and required more studies. The findings of our study also gave a new insight into the onset of CLE. The NOD-like receptor signaling pathway might provide a new therapeutic target pathway of CLE. Owing that our study is only a bioinformatics study, our results require further validation.

## Figures and Tables

**Figure 1:** Identification of DEGs via volcano plot analysis.

**Figure 2:** Authentication of 176 commonly DEGs of SCLE in two datasets (GSE109248 and GSE113942) through Venn diagram software.

**Figure 3:** GO enrichment and KEGG analysis of DEGs in SCLE and CCLE (upper: CCLE; lower: SCLE; left: bubble charts; right: column charts).

**Figure 4:** (a) Common DEG PPI network of SCLE conducted by STRING online database and (b) top 10 genes identified by Cytohubba.

**Figure 5:** (a) Common DEG PPI network of CCLE conducted by STRING online database and (b) top 10 genes identified by Cytohubba.

**Table 1:** Gene ontology and KEGG analysis of DEGs in CCLE.

Ontology	ID	Description	GeneRatio	BgRatio	*P* value	Adjusted *P*	*q* value
BP	GO:0009615	Response to virus	50/261	326/18670	1.70*e* − 37	5.24*e* − 34	4.00*e* − 34
BP	GO:0051607	Defense response to virus	44/261	238/18670	1.22*e* − 36	1.88*e* − 33	1.44*e* − 33
BP	GO:0043900	Regulation of multiorganism process	40/261	405/18670	1.35*e* − 22	1.39*e* − 19	1.06*e* − 19
BP	GO:0048525	Negative regulation of viral process	23/261	99/18670	6.22*e* − 22	4.80*e* − 19	3.66*e* − 19
BP	GO:0051249	Regulation of lymphocyte activation	40/261	485/18670	9.92*e* − 20	5.42*e* − 17	4.13*e* − 17
CC	GO:0009897	External side of plasma membrane	31/270	393/19717	3.76*e* − 15	1.06*e* − 12	9.91*e* − 13
CC	GO:0001533	Cornified envelope	7/270	65/19717	2.95*e* − 05	0.004	0.004
CC	GO:0030667	Secretory granule membrane	12/270	298/19717	8.77*e* − 04	0.082	0.077
MF	GO:0042379	Chemokine receptor binding	10/257	66/17697	3.62*e* − 08	9.06*e* − 06	7.84*e* − 06
MF	GO:0005126	Cytokine receptor binding	19/257	286/17697	4.08*e* − 08	9.06*e* − 06	7.84*e* − 06
MF	GO:0042287	MHC protein binding	8/257	40/17697	9.13*e* − 08	1.35*e* − 05	1.17*e* − 05
MF	GO:0005125	Cytokine activity	16/257	220/17697	1.44*e* − 07	1.47*e* − 05	1.27*e* − 05
MF	GO:0048020	CCR chemokine receptor binding	8/257	43/17697	1.66*e* − 07	1.47*e* − 05	1.27*e* − 05
KEGG	hsa04060	Cytokine-cytokine receptor interaction	28/143	295/8076	1.59*e* − 13	3.01*e* − 11	2.41*e* − 11
KEGG	hsa04061	Viral protein interaction with cytokine and cytokine receptor	15/143	100/8076	1.76*e* − 10	1.67*e* − 08	1.34*e* − 08
KEGG	hsa05340	Primary immunodeficiency	10/143	38/8076	6.84*e* − 10	4.31*e* − 08	3.46*e* − 08
KEGG	hsa04621	NOD-like receptor signaling pathway	18/143	181/8076	2.44*e* − 09	1.15*e* − 07	9.26*e* − 08
KEGG	hsa04640	Hematopoietic cell lineage	12/143	99/8076	1.48*e* − 07	5.59*e* − 06	4.48*e* − 06

**Table 2:** Gene ontology and KEGG analysis of DEGs in SCLE.

Ontology	ID	Description	GeneRatio	BgRatio	*P* value	Adjusted *P*	*q* value
BP	GO:0009615	Response to virus	25/154	326/18670	2.36*e* − 17	5.70*e* − 14	4.86*e* − 14
BP	GO:0051607	Defense response to virus	22/154	238/18670	4.37*e* − 17	5.70*e* − 14	4.86*e* − 14
BP	GO:0034341	Response to interferon-gamma	18/154	199/18670	5.40*e* − 14	4.69*e* − 11	4.00*e* − 11
BP	GO:0071346	Cellular response to interferon-gamma	17/154	180/18670	1.38*e* − 13	8.99*e* − 11	7.67*e* − 11
BP	GO:0060337	Type I interferon signaling pathway	12/154	95/18670	1.95*e* − 11	8.49*e* − 09	7.24*e* − 09
MF	GO:0042288	MHC class I protein binding	4/153	20/17697	2.34*e* − 05	0.009	0.008
MF	GO:0008009	Chemokine activity	5/153	49/17697	6.35*e* − 05	0.012	0.011
MF	GO:0042379	Chemokine receptor binding	5/153	66/17697	2.64*e* − 04	0.033	0.030
MF	GO:0042287	MHC protein binding	4/153	40/17697	3.85*e* − 04	0.036	0.033
KEGG	hsa04060	Cytokine-cytokine receptor interaction	11/84	295/8076	2.21*e* − 04	0.023	0.022
KEGG	hsa05164	Influenza A	8/84	171/8076	3.80*e* − 04	0.023	0.022
KEGG	hsa04623	Cytosolic DNA-sensing pathway	5/84	63/8076	4.73*e* − 04	0.023	0.022
KEGG	hsa04621	NOD-like receptor signaling pathway	8/84	181/8076	5.56*e* − 04	0.023	0.022
KEGG	hsa04061	Viral protein interaction with cytokine and cytokine receptor	6/84	100/8076	5.78*e* − 04	0.023	0.022

**Table 3:** The top hub genes of SCLE.

Gene symbol	Description	Degree of connectivity
STAT1	Signal transducer and activator of transcription 1	88
CXCL10	C-X-C motif chemokine ligand 10	78
IRF7	Interferon regulatory factor 7	70
ISG15	ISG15 ubiquitin-like modifier	68
RSAD2	Radical S-adenosyl methionine domain-containing 2	64
IFIT3	Interferon-induced protein with tetratricopeptide repeats 3	64
OASL	2′-5′-Oligoadenylate synthetase like	62
GBP1	Guanylate-binding protein 1	62
OAS1	2′-5′-Oligoadenylate synthetase 1	60
OAS2	2′-5′-Oligoadenylate synthetase 2	60

**Table 4:** The top hub genes of CCLE.

Gene symbol	Description	Degree of connectivity
CXCL10	C-X-C motif chemokine ligand 10	60
IRF7	Interferon regulatory factor 7	56
IFIT3	Interferon-induced protein with tetratricopeptide repeats 3	54
CTLA4	Cytotoxic T lymphocyte-associated protein 4	50
ISG15	ISG15 ubiquitin-like modifier	50
OAS2	2′-5′-Oligoadenylate synthetase 2	50
RASD2	Radical S-adenosyl methionine domain-containing 2	48
CCL5	C-C motif chemokine ligand 5	48
GBP1	Guanylate-binding protein 1	46
OAS1	2′-5′-Oligoadenylate synthetase 1	46

## Data Availability

The datasets generated and/or analyzed during the current study are available in the GSE109248 repository (https://www.ncbi.nlm.nih.gov/geo/query/acc.cgi?acc=GSE109248) and in the GSE112943 repository (https://www.ncbi.nlm.nih.gov/geo/query/acc.cgi?acc=GSE112943).

## References

[1] Jonsson R., Heyden G., Westberg N. G., Nyberg G. (1984). Oral mucosal lesions in systemic lupus erythematosus - a clinical, histopathological and immunopathological study. *The Journal of Rheumatology*.

[2] Burge S. M., Frith P. A., Juniper R. P., Wojnarowska F. (1989). Mucosal involvement in systemic and chronic cutaneous lupus erythematosus. *British Journal of Dermatology*.

[3] Del Barrio-Diaz P., Reyes-Vivanco C., Cifuentes-Mutinelli M., Manriquez J., Vera-Kellet C. (2020). Association between oral lesions and disease activity in lupus erythematosus. *Journal of the European Academy of Dermatology*.

[4] Stannard J. N., Kahlenberg J. M. (2016). Cutaneous lupus erythematosus: updates on pathogenesis and associations with systemic lupus. *Current Opinion in Rheumatology*.

[5] Hejazi E. Z., Werth V. P. (2016). Cutaneous lupus erythematosus: an update on pathogenesis, diagnosis and treatment. *American Journal of Clinical Dermatology*.

[6] Wenzel J., Uerlich M., Rrenk W. (2005). Scarring skin lesions of discoid lupus erythematosus are characterized by high numbers of skin-homing cytotoxic lymphocytes associated with strong expression of the type I interferon-induced protein MxA. *Blackwell Science Ltd*.

[7] Wenzel J. (2019). Cutaneous lupus erythematosus: new insights into pathogenesis and therapeutic strategies. *Nature Reviews Rheumatology*.

[8] Scholtissek B., Zahn S., Maier J. (2017). Immunostimulatory endogenous nucleic acids drive the lesional inflammation in cutaneous lupus erythematosus. *The Journal of Investigative Dermatology*.

[9] Sarkar M. K., Hile G. A., Tsoi L. C. (2018). Photosensitivity and type I IFN responses in cutaneous lupus are driven by epidermal-derived interferon kappa. *Annals of the Rheumatic Diseases*.

[10] Ko W., Li L., Young T. R. (2021). Gene expression profiling in the skin reveals strong similarities between subacute and chronic cutaneous lupus that are distinct from lupus nephritis. *The Journal of Investigative Dermatology*.

[11] Meltzer D. P. S. (2007). GEOquery: a bridge between the Gene Expression Omnibus (GEO) and BioConductor. *Bioinformatics*.

[12] Sontheimer R. D. (2005). Subacute cutaneous lupus erythematosus: 25-year evolution of a prototypic subset (subphenotype) of lupus erythematosus defined by characteristic cutaneous, pathological, immunological, and genetic findings. *Autoimmunity Reviews*.

[13] Chong B. F., Song J., Olsen N. J. (2012). Determining risk factors for developing systemic lupus erythematosus in patients with discoid lupus erythematosus. *British Journal of Dermatology*.

[14] Gallucci S., Meka S., Gamero A. M. (2021). Abnormalities of the type I interferon signaling pathway in lupus autoimmunity. *Cytokine*.

[15] Wenzel J., Zahn S., Mikus S., Wiechert A., Bieber T., Tüting T. (2007). The expression pattern of interferon-inducible proteins reflects the characteristic histological distribution of infiltrating immune cells in different cutaneous lupus erythematosus subsets. *The British Journal of Dermatology*.

[16] Wenzel J., Wrenkmper E., Freutel S., Henze S., Tüting T. (2010). Enhanced type I interferon signalling promotes Th1-biased inflammation in cutaneous lupus erythematosus. *The Journal of Pathology*.

[17] Nico M., Vilela M. A. C., Rivitti E. A., Loureno S. V. (2008). Oral lesions in lupus erythematosus: correlation with cutaneous lesions. *European Journal of Dermatology*.

[18] (2010). Oral lesions in lupus erythematosus–cytokines profiles of inflammatory infiltrate. *Journal of Cutaneous Pathology*.

[19] Baechler E. C., Batliwalla F. M., Karypis G. (2003). Interferon-inducible gene expression signature in peripheral blood cells of patients with severe lupus. *Proceedings of the National Academy of Sciences of the United States of America*.

[20] Yuan Y., Ma H., Ye Z., Jing W., Jiang Z. (2018). Interferon-stimulated gene 15 expression in systemic lupus erythematosus. *Zeitschrift für Rheumatologie*.

[21] Braunstein I., Klein R., Okawa J., Werth V. P. (2012). The interferon-regulated gene signature is elevated in subacute cutaneous lupus erythematosus and discoid lupus erythematosus and correlates with the cutaneous lupus area and severity index score. *The British Journal of Dermatology*.

[22] Fu Q., Zhao J., Qian X. (2011). Association of a functional IRF7 variant with systemic lupus erythematosus. *Arthritis & Rheumatism*.

[23] Fang W., Zou Y. F., Sun G. P. (2011). Association between functionalIRF7variant and systemic lupus erythematosus may need more critical examination: comment on the article by Fu et al. *Arthritis & Rhematology*.

[24] Tanya S., Artem V., Sadik C. D., Detlef Z., Yask G., Ludwig R. J. (2018). Gene expression analysis reveals novel shared gene signatures and candidate molecular mechanisms between pemphigus and systemic lupus erythematosus in CD4+ T cells. *Frontiers in Immunology*.

[25] Fan H., Zhao G., Ren D., Liu F., Dong G., Hou Y. (2017). Gender differences of B cell signature related to estrogen-induced IFI44L/BAFF in systemic lupus erythematosus. *Immunology Letters*.

[26] Liu W., Li M., Wang Z., Wang J. (2020). IFN-*γ* mediates the development of systemic lupus erythematosus. *BioMed Research International*.

[27] Wang J., Dai M., Cui Y. (2018). Association of abnormal elevations in IFIT3 with overactive cyclic GMP-AMP synthase/stimulator of interferon genes signaling in human systemic lupus erythematosus monocytes. *Rheumatology*.

[28] Méndez-Flores S., Hernández-Molina G., Azamar-Llamas D., Zúñiga J., Romero-Díaz J., Furuzawa-Carballeda J. (2019). Inflammatory chemokine profiles and their correlations with effector CD4 T cell and regulatory cell subpopulations in cutaneous lupus erythematosus. *Cytokine*.

[29] Chen L., Cao S. Q., Lin Z. M., He S. J., Zuo J. P. (2021). NOD-like receptors in autoimmune diseases. *Acta Pharmacologica Sinica*.

[30] Yu S. L., Wong C. K., Wong P. T. Y. (2011). Down-regulated NOD2 by immunosuppressants in peripheral blood cells in patients with SLE reduces the muramyl dipeptide-induced IL-10 production. *PLoS One*.

